The article "A Chaperonin Subunit with Unique Structures Is Essential for Folding of a Specific Substrate" was retracted in 2022. Reasons: fabricated or falsified data; fabricated or falsified images; an official misconduct investigation; misconduct by an author.

# A Chaperonin Subunit with Unique Structures Is Essential for Folding of a Specific Substrate

**DOI:** 10.1371/journal.pbio.1001040

**Published:** 2011-04-05

**Authors:** Lianwei Peng, Yoichiro Fukao, Fumiyoshi Myouga, Reiko Motohashi, Kazuo Shinozaki, Toshiharu Shikanai

**Affiliations:** 1 Department of Botany, Graduate School of Science, Kyoto University, Sakyo-ku, Kyoto, Japan; 2 Plant Global Educational Project, Graduate School of Biological Sciences, Nara Institute of Science and Technology, Takayama, Ikoma, Nara, Japan; 3 Gene Discovery Research Group, RIKEN Plant Science Center, Yokohama, Japan; 4 Faculty of Agriculture, University of Shizuoka, Shizuoka, Japan; Yale School of Medicine/HHMI, United States of America

## Abstract

Type I chaperonins are large, double-ring complexes present in bacteria (GroEL), mitochondria (Hsp60), and chloroplasts (Cpn60), which are involved in mediating the folding of newly synthesized, translocated, or stress-denatured proteins. In *Escherichia coli*, GroEL comprises 14 identical subunits and has been exquisitely optimized to fold its broad range of substrates. However, multiple Cpn60 subunits with different expression profiles have evolved in chloroplasts. Here, we show that, in *Arabidopsis thaliana*, the minor subunit Cpn60β4 forms a heterooligomeric Cpn60 complex with Cpn60α1 and Cpn60β1–β3 and is specifically required for the folding of NdhH, a subunit of the chloroplast NADH dehydrogenase-like complex (NDH). Other Cpn60β subunits cannot complement the function of Cpn60β4. Furthermore, the unique C-terminus of Cpn60β4 is required for the full activity of the unique Cpn60 complex containing Cpn60β4 for folding of NdhH. Our findings suggest that this unusual kind of subunit enables the Cpn60 complex to assist the folding of some particular substrates, whereas other dominant Cpn60 subunits maintain a housekeeping chaperonin function by facilitating the folding of other obligate substrates.

## Author Summary

Chaperonins assist the folding of some nascent and denatured proteins to their native, functional forms. Each chaperonin consists of a pair of protein complexes resembling two stacked toroids; folding occurs inside the toroid cavity. Chaperonins are ubiquitous in both bacteria and more complex nucleated cells, as well as in the intracellular organelles that have evolved from bacteria by endosymbiosis: mitochondria and, in plants, chloroplasts. They are indispensable for cellular function. Many different chaperonin subunits have evolved in various species of bacteria as well as in most mitochondria and chloroplasts. The physiological and functional relevance of these multiple chaperonin subunits is poorly understood, however. In this study, we have characterized the minor chaperonin subunit Cpn60β4 from *Arabidopsis* chloroplasts, which differs in structure from other chloroplast chaperonins. When the *Cpn60β4* gene is defective, the plants fail to accumulate one protein complex in particular: the chloroplast NADH dehydrogenase-like complex (NDH). We discovered that Cpn60β4 forms a complex with other Cpn60 α and *β* subunits and that this complex is essential for the folding of the NDH subunit NdhH. Cpn60β4 has a unique protein “tail” that is required for the efficient folding of NdhH. Our findings suggest that Cpn60β4 has evolved with distinctive structural features that facilitate the folding of one specific substrate and that this strategy is used by plants to satisfy their conflicting requirements for chaperonins with both specialized and general functions.

## Introduction

Chaperonins are large double-ring assemblies that assist in the efficient folding of substrate proteins (reviewed in [1]–[3]). Two types of chaperonins have been identified: type I in bacteria (GroEL), mitochondria (Hsp60), and chloroplasts (Cpn60), and type II in archaea (thermosome) and eukaryotic (TRiC/CCT) cytosol (reviewed in [4]). Whereas a type I chaperonin ring is composed of seven subunits, a type II chaperonin ring consists of eight or nine subunits that are not identical but are homologous. Type I chaperonin requires co-chaperonin GroES/Hsp10 for substrate encapsulation, whereas type II chaperonin is independent of GroES/Hsp10 factors. Both types of chaperonins utilize ATP as energy to drive a series of structural rearrangements that allow them to capture, encapsulate, and release the substrate proteins (reviewed in [4]).

The GroEL/GroES complex from *Escherichia coli* (*E. coli*) represents the type I chaperonins and its structure and function have been studied extensively (reviewed in [4],[5]). GroEL consists of 14 identical subunits of ∼57 kDa and these subunits form two heptameric rings stacked back-to-back with a central cavity in each ring [6]. Each subunit contains three domains. An equatorial domain comprises the ATP/ADP binding site and an apical domain contains the hydrophobic surface toward the ring cavity for polypeptide binding. The intermediate domain links the equatorial and apical domains [6],[7]. The co-chaperonin GroES is a homoheptameric single-ring composed of 10 kDa subunits [8]. GroES can rapidly bind the substrate-captured GroEL ring (*cis* ring) in the presence of ATP; hence, the GroEL/GroES complex provides an encapsulated cavity for protein folding [9],[10]. Due to structural rearrangements in the apical and intermediate domains, the *cis* cavity becomes enlarged and the physical features of the cavity wall change. This process lasts about 10–15 s and is accompanied by the hydrolysis of seven ATP molecules. After hydrolysis, ATP and other non-native peptides bind to the GroEL in the *trans* ring, triggering dissociation of the GroES from the opposite ring. The folded protein is then released from the chaperonin complex (reviewed in [1]–[5]).

Proteome-wide analysis of chaperonin-dependent protein folding has shown that GroEL interacts with about 250 different proteins and these substrates are categorized into three classes [11]. The class I substrates are independent of GroEL/GroES, whereas class II substrates are partially dependent on GroEL/GroES, and they can utilize other chaperone systems, such as DnaK, for folding. A total of 84 proteins are grouped into class III and they are potential obligate substrates of GroEL/GroES in vivo [11]. More recently, Fujiwara et al. [12] employed a more direct approach by testing the solubility of class III substrates in GroE-depleted cells and found that only ∼60% (49 out of 84) of the class III proteins are absolutely dependent on GroEL/GroES for folding. Furthermore, an additional eight proteins that were not identified as class III proteins were also found to be GroEL/GroES obligate substrates and the authors defined these 57 proteins as class IV obligate substrates [12]. The majority of the class IV proteins are involved in metabolic reactions. Bioinformatic analysis has shown that nearly half of the class IV proteins contain TIM-barrel folds. In addition to these TIM-barrel folds, FAD/NAD(P)-binding domains, PLP-dependent transferase-like folds, and thiolase folds are also highly enriched in the group [12]. These data suggest that GroEL/GroES has been optimized to facilitate the folding of a variety of substrates during evolution.

The basic features of the mechanisms for GroEL/GroES-mediated folding of the nonnative substrates have been demonstrated by a great number of functional and structural studies. However, these studies have focused primarily on the model chaperonin system that is composed of uniform subunits, such as GroEL from *E. coli*. In contrast to *E. coli*, nearly 30% of bacterial genomes contain two or more chaperonin genes [13]. Furthermore, almost all mitochondria and chloroplasts studied in higher plants possess multiple chaperonin subunits [14]. There have been few reports focusing on the role played by multiple chaperonin genes. In *Sinorhizobium meliloti*, one of the five GroEL paralogs, GroEL1 was shown to be required for NodD protein folding [15]. However, overexpression of another GroEL protein can suppress the defect of the *groEL1* mutant [15]. There are similar reports in other bacteria; *Bradyrhizobium japonicum* possesses at least five highly conserved *groESL* operons. Although nitrogen fixation activity was reduced to approximately 5% of the wild-type (WT) level in the double mutant defective in *groEL3* and *groEL4*, overexpression of two of the other *groESL* operons partially suppressed this phenotype [16]. Of the three chaperonin genes of *Rhizobium leguminosarum*, only *Cpn60.1* is essential for growth. Overexpression of the *Cpn60.3* gene in the *cpn60.1* mutant sustains bacterial growth, but the complemented strain is sensitive to high temperature, suggesting that Cpn60.3 does not facilitate the folding of particular proteins supporting the growth of bacteria at high temperature [17]. By contrast, the specificity of GroEL1 function in *Mycobacterium smegmatis* seems to be absolute. This chaperonin is not essential for growth but is required for mycolic acid biosynthesis during mature biofilm formation [18]. GroEL1 may be specifically involved in the folding of two proteins, KasA and SmEG4308, which are required for mycolic acid synthesis, or in converting KasA between two isoforms [18]. These lines of evidence suggest that the functions of the multiple chaperonin subunits are specialized, although they have different degrees of specificity.

Chloroplast type I chaperonin complex (Cpn60) is similar in structure to GroEL and also consists of two stacked heptameric rings [19],[20]. In contrast to GroEL, which is composed of identical subunits, Cpn60 comprises two different subunit types, Cpn60α and Cpn60β [21]–[23], and they are only approximately 50% identical to each other [14]. In vitro reconstitution studies of the chloroplast Cpn60 complex suggested a stoichiometry of α7β7 in the Cpn60 complex [24], which is in accordance with the observation that roughly equal amounts of α and β subunits are present in chaperonin oligomers purified from spinach chloroplasts [25]. However, it is still unclear how these subunits are organized within a complex. Furthermore, the *Arabidopsis thaliana* genome contains two genes encoding Cpn60α subunits and four genes encoding Cpn60β subunits [14], and they have different expression profiles [26],[27]. Cpn60α1 (At2g28000), Cpn60β1 (At1g55490), and Cpn60β2 (At3g13470) are the dominant Cpn60 subunits, whereas Cpn60α2 (At5g18820), Cpn60β3 (At5g56500), and Cpn60β4 (At1g26230) are present at very low levels. Disruption of the *Cpn60α1* gene results in general defects in plastid function, leading to embryonic lethality [28], which highlights the critical role of Cpn60α1 in maintaining plastid function. The *cpn60β1β2* double mutant also shows the lethal phenotype [29], suggesting that Cpn60α1 and Cpn60β1–β2 form a heterooligomer that provides the housekeeping chaperonin function in chloroplasts by assisting the folding of a wide range of proteins.

Multiple subunits also occur in type II chaperonin CCT and certain subunits are responsible for the binding of specific substrates, such as actin and tubulin [30]. Recently, it has been suggested that different subunits of CCT play unique roles in determining substrate specificity [31]. However, few reports have focused on the function of the multiple subunits in the chloroplast chaperonin system. In particular, whereas the amino acid sequences of the Cpn60β1–β3 subunits share 90%–95% identity, Cpn60β4 is only 60% identical to each of the other three Cpn60β subunits [14]. So far, there has been no explanation why plants evolved this unusual kind of Cpn60β subunit. In this study, we showed that Cpn60β4 is strictly and specifically required for the folding of the NdhH protein, a subunit of the chloroplast NADH dehydrogenase-like complex (NDH).

## Results

### The *Arabidopsis crr27* Mutant Is Specifically Defective in NDH Activity

NDH is a multi-subunit complex embedded in the thylakoid membrane and is involved in chlororespiration and photosystem I (PSI) cyclic electron transport (Figure 1A) [32]. The activity of NDH can be monitored as a post-illumination rise in chlorophyll fluorescence (Figure 1B) due to reduction of the plastoquinone (PQ) pool by the NDH complex in the dark [33]. Based on this phenomenon, we isolated dozens of *Arabidopsis* mutants specifically defective in NDH activity, which we referred to as *chlororespiratory reduction* (*crr*) mutants. Characterization of these mutants led to the identification of several NDH subunits and a large body of proteins involved in the expression of subunit genes and the assembly or stabilization of the NDH complex (reviewed in [34],[35]). Here, we identify two mutants, *cpn60α1* and *crr27*, neither of which showed the increase in fluorescence after actinic light (AL) illumination, indicating impaired NDH activity (Figure 1B). In contrast to *crr* mutants, the *cpn60α1* mutant exhibited retarded growth and pale green-leaf phenotypes (Figure 1C). Map-based cloning identified a single amino acid substitution (D335A) at a conserved position in *cpn60α1* (Figure 1D). Although the total levels of Cpn60α and Cpn60β were increased in *cpn60α1*, possibly due to complementation effects, the levels of many other chloroplast proteins, including NDH subunits, were reduced to various extents (Figure S1), supporting the idea that Cpn60 has a diverse set of substrates. The reduction in NDH (25%–50%) in *cpn60α1* at least partly explains the failure to detect NDH activity by chlorophyll fluorescence.

**Figure 1:** Characterization of *cpn60α1* and *crr27* mutants. (A) A schematic model of NDH function. The NDH complex mediates electron transfer from the stromal reducing pool to plastoquinone (PQ). PQ reduction in the dark depends on NDH activity and can be detected by the transient rise of chlorophyll (Chl) fluorescence after illumination with actinic light (AL). For simplicity, this model does not include the information that NDH interacts with PSI. Cyt, cytochrome; PC, plastocyanin; Fd, ferredoxin. (B) Determination of NDH activity using Chl fluorescence analysis. The bottom curve indicates a typical trace of Chl fluorescence in the WT plants. Leaves were exposed to AL for 5 min. AL was turned off and the subsequent transient rise in fluorescence ascribed to NDH activity was monitored using a PAM Chl fluorometer. Insets are magnified traces from the boxed area. *crr27-1+Cpn60β4* and *crr27-1+Cpn60β4-HA* represent *crr27-1* transformed by the WT genomic *Cpn60β4* and genomic *Cpn60β4* fused to the HA epitope-tag, respectively. *crr27-1+35S::Cpn60β4-HA* and *crr27-1+35S::Cpn60β1-HA* represent *crr27-1* transformed with Cpn60β4 and Cpn60β1 cDNA, respectively, fused to the sequence encoding the HA-tag expressed under the control of the CaMV *35S* promoter. Fluorescence levels were standardized to the maximum fluorescence levels of closed PSII (*Fm*) by applying saturating-light pulses (SP). ML, measuring light; *Fo*, minimum fluorescence level of open PSII. (C) Visible phenotype of mutants. Seedlings were cultured at 50 µmol photons m^−2^ s^−1^ for 4 wk after germination. (D and E) Mutations in *cpn60α1* (D) and three *crr27* mutant alleles (E) are indicated. (F) RT-PCR analysis of the *Cpn60β4* transcript in WT and *crr27* mutants. *ACT8* was used as a control.

The *crr27* mutants were isolated by screening *Ds* transposon-tagged lines using PAM (pulse amplitude modulation) fluorometry [36],[37]. Unlike *cpn60α1*, *crr27* mutants did not exhibit any visible phenotype besides impaired NDH activity (Figure 1B and 1C). The *Cpn60β4* gene was knocked out by *Ds* or T-DNA insertions in three *crr27* alleles, and reverse transcription (RT)-PCR analysis did not detect any *Cpn60β4* transcripts (Figure 1E and 1F). Full NDH activity was rescued by the introduction of the WT *Cpn60β4* gene into *crr27-1* (Figure 1B). Two chlorophyll fluorescence parameters, ETR (electron transport rate) and NPQ (nonphotochemical quenching), indicate subtle defects in photosynthesis and are therefore often used to characterize mutants with defective photosynthetic apparatus. ETR was only slightly reduced and NPQ was not affected in *crr27-1* (Figure S2), which is consistent with the phenotypes of other *crr* mutants with specific defects in NDH activity.

### Accumulation of NDH Subcomplex Is Impaired in the Absence of Cpn60β4

NDH interacts with at least two copies of PSI to form the NDH-PSI supercomplex (Figure 2A) [35], which can be separated by blue native (BN)-PAGE [38],[39]. To study the role of Cpn60β4 in biogenesis of the NDH complex, thylakoid protein complexes from WT and *crr27* mutants were separated by BN-PAGE. No difference was found in the major complex bands between WT and *crr27* (Figures 2B and S3A). However, band I, corresponding to the NDH-PSI supercomplex detected in WT, was replaced by band II, corresponding to the subsupercomplex in *crr27,* as in the NdhL-defective *ndhl (crr23)* mutant (Figure 2B) [38]. Based on extensive genetic and biochemical characterizations, we divided the NDH complex into four categories: membrane, lumen, and A and B subcomplexes (Figure 2A) [39]. Previous mass analysis revealed that only subcomplex A, which is composed of four plastid-encoded subunits (NdhH–NdhK) and four nucleus-encoded subunits (NdhL–NdhO), was absent in band II (Figure 2A) [39]. Immunoblot analysis confirmed that the levels of subcomplex A subunits NdhH and NdhL were dramatically decreased in *crr27,* whereas subunits of the other NDH subcomplexes, NDH18, NDF1, and FKBP16-2, were only slightly reduced (Figure 2C). Consistent with the invisible growth phenotype of *crr27*, identical levels of D1 (PSII complex), PsaA (PSI complex), and cytochrome (Cyt) *f* (Cyt *b*_6_ *f* complex) were detected in *crr27* and WT (Figure 2C). In addition, no significant difference in stromal protein levels was detected between WT and *crr27-1* mutants by clear native (CN)-PAGE and subsequent two-dimensional (2D)/SDS-PAGE (Figure S3B). From these results, we conclude that the accumulation of NDH subcomplex A was specifically impaired in the absence of Cpn60β4.

**Figure 2:** Accumulation of NDH subcomplex A was impaired in *crr27*. (A) A schematic model of the NDH-PSI supercomplex in chloroplasts. The NDH complex is divided into four subcomplexes and interacts with at least two copies of PSI to form the NDH-PSI supercomplex corresponding to Band I, which can be detected by BN-PAGE (B). Eleven plastid-encoded subunits are depicted by green letters; nucleus-encoded subunits are depicted by red letters. Subcomplex A, surrounded by the red line, is missing in the sub-NDH-PSI supercomplex corresponding to Band II, which is detected in *crr27* and *ndhl* mutants (B). (B) BN-PAGE analysis of thylakoid protein complexes. After electrophoresis**,** the gel was stained with CBB. The complexes are identified in the original non-stained gel in Figure S3A. (C) Immunoblot analysis of the thylakoid proteins from various genetic backgrounds with the indicated antibodies. Thylakoid proteins were loaded on an equal chlorophyll basis, and the series of dilutions is indicated.

### Heterooligomeric Chaperonin Complex Formation of Cpn60β4 with Cpn60β1–β3 and Cpn60α1

Previous transcriptomic analysis [26] indicated that the expression level of the *Cpn60β* *4* gene is lower than that of other *Cpn60β* genes. Furthermore, the Cpn60β4 subunit could not be visualized with Coomassie Brilliant Blue (CBB) staining in the 2D CN/SDS-PAGE gel, whereas other Cpn60β subunits and Cpn60α1 were detected [27], suggesting that the stoichiometry of Cpn60β4 is extremely low compared to the other Cpn60β subunits. To confirm the accumulation of Cpn60β4 in WT, we separated total stromal protein complexes isolated from WT plants by CN-PAGE. The protein band corresponding to the position of the Cpn60 complex was excised from the gel (Figure S4A) and analyzed by liquid chromatography-tandem mass spectrometry (LC-MS/MS) analysis using the linear ion-trap triple quadrupole (LTQ)-Orbitrap XL-HTC-PAL system, which provides high mass accuracy, high resolution, and high sensitivity. The values of Mowse score, Protein match, and emPAI (exponentially modified Protein Abundance Index) are commonly used to estimate relative protein levels. LC-MS/MS analyses detected the Cpn60β4 protein, but its level was significantly lower than those of the other three Cpn60β proteins (Figure S4B; Table S1). Consistent with the apparent mutant phenotype (Figures 1 and 2), we confirmed the accumulation of Cpn60β4 in WT (Figure S4C).

In contrast to *cpn60α1*, the *crr27* mutation did not affect total Cpn60α or Cpn60β levels (Figures 3A and S1A). To study the role of Cpn60β4, a chimeric gene encoding an HA (influenza hemagglutinin protein epitope) tag fused to the C-terminus of Cpn60β4 was introduced into *crr27-1*. This transformation fully restored NDH activity (Figure 1B), indicating that the HA-tag did not affect the function of Cpn60β4. We also overexpressed HA-tagged Cpn60β1 and Cpn60β4 in *crr27-1* under control of the cauliflower mosaic virus (CaMV) *35S* promoter. NDH activity and NDH subcomplex A level were rescued only in the *35S::Cpn60β4-HA* lines (Figures 1B and 2C), indicating that Cpn60β1 cannot complement the function of Cpn60β4, even under the control of the same promoter.

**Figure 3:** Analysis of the Cpn60β4 subunit. (A) Cpn60β4 is localized to the chloroplast stroma. Freshly isolated chloroplasts from various genotypes were separated into membrane and stromal fractions. Immunoblot analysis was performed using the indicated antibodies. RbcL and Cyt *f* were detected as loading and fractionation controls. (B) Stromal protein complexes isolated from *crr27-1* complemented by Cpn60β4-HA were separated by CN-PAGE, followed by 2-dimensional SDS-PAGE. The proteins were immunodetected with specific antibodies. A short arrow indicates the position of the Cpn60 complex. (C) Heterooligomeric complex formation between Cpn60β4, Cpn60α1, and Cpn60β1–β3. Chaperonin complex containing Cpn60β4 was purified from the *crr27-1* mutant plants expressing HA-tagged Cpn60β4 using the µMACS HA isolation kit. After elution, total proteins were separated by 7.5% SDS-PAGE and stained with CBB. The signals were quantitatively analyzed with Imagemaster software (Amersham Pharmacia Biotech). The stoichiometry of Cpn60β4, Cpn60β1–β3, and Cpn60α1 in the specific chaperonin complex containing Cpn60β4 was estimated to be 17:37:46 and 14:39:47 in the two independent purifications (E1 and E2), respectively.

Cpn60β4 localized to the chloroplast stroma (Figure 3A) and co-migrated with other Cpn60β and Cpn60α subunits in CN-PAGE (Figures 3B and S4), suggesting that Cpn60β4 is an intrinsic subunit of the Cpn60 complex. To examine this possibility, HA-tagged Cpn60β4 was enriched from the stromal fraction isolated from *crr27-1* plants complemented with Cpn60β4-HA using the µMACS HA isolation kit (Miltenyi Biotec) under previously established conditions [11]. Because the additional HA tag in the C-terminus does not affect the function of Cpn60β4 (Figure 1B), their interacting proteins might also be co-purified. Total isolated proteins were separated by SDS-PAGE (Figure S5A) and further analyzed by LC-MS/MS analysis. Both Cpn60α1 and Cpn60β1–β4 subunits were detected in the purified sample and MS analysis showed that they were the most abundant proteins (Tables 1 and S2), implying that Cpn60β4 forms a specific heterooligomeric Cpn60 complex with Cpn60α1 and other Cpn60β subunits.

**Table 1:** Summary of the chaperonin and NDH subunits detected in the Cpn60β1 and Cpn60β4 IP fractions.

Protein Name		Cpn60β1 IP			Cpn60β4 IP		emPAI Ratio^a^
	Mowse Score	Protein Match	Coverage (%)	Mowse Score	Protein Match	Coverage (%)	
Cpn60α1	2,177	64	69	6,369	188	72	3.9
Cpn60β1	6,794	230	70	5,591	202	68	0.47
Cpn60β2	5,689	178	59	5,356	182	67	0.87
Cpn60β3	3,624	119	36	3,448	123	37	1.26
Cpn60β4	226^b^	13^b^	3^b^	3,348	156	74	101
NdhJ	57	2	15	—	—	—	—
NdhH	44	2	4	614	24	53	43.4

a. emPAI Ratio means the ratio between emPAI score of proteins isolated from Cpn60β4 IP and Cpn60β1 IP fraction.

b. The sequences of these 13 peptides are identical between Cpn60β1 and Cpn60β4, suggesting that they are sequenced from Cpn60β1. RT-PCR showed that *crr27-1* is a null mutant (Figure 1F).

The molecular masses of Cpn60β4-HA, Cpn60β1–β3, and Cpn60α1 are 64.4, 58.2, and 57.1 kDa, respectively, which enables us to distinguish them in SDS-PAGE. The purified proteins were subjected to 7.5% SDS-PAGE and three major bands with molecular masses of approximately 60 kDa were visualized with CBB staining (Figure 3C). Based on the mobility, three bands should correspond to Cpn60β4-HA, Cpn60β1–β3, and Cpn60α1 (Figure 3C). Quantitative estimation of these signals showed that the level of Cpn60α1 is about 50% of all of the chaperonin subunits, which is consistent with the proposal that the Cpn60 complex is composed in a α7β7 stoichiometry [24],[25]. However, the level of Cpn60β4 in the chaperonin complex was lower (∼15%) (Figure 3C), implying that approximately two molecules of Cpn60β4 are included in double rings, as well as five molecules of other Cpn60β subunits. Based on the stoichiometry of the Cpn60β4 subunit in total Cpn60 subunits [26],[27], the majority of the Cpn60 complex is unlikely to contain Cpn60β4, and we estimated its stoichiometry in the specific complex including Cpn60β4.

### NdhH Is Specifically Associated with Cpn60β4

Given that Cpn60β4 is an intrinsic subunit of the chaperonin complex (Figure 3) and that the NDH subcomplex A was missing in the *crr27* mutants (Figure 2), it is very likely that the specific chaperonin complex containing Cpn60β4 is required for the folding of at least one subunit of the NDH subcomplex A. If this is the case, the interacting NDH subunit would be copurified with Cpn60β4-HA. To determine differences in substrate specificity, protein complexes containing Cpn60β1 were isolated using the *35S::Cpn60β1-HA* lines. Neither Cpn60 nor NDH subunits were detected in untransformed WT plants, which were used as a negative control (Figure S5A; Table S2), excluding the possibility of non-specific binding to the magnetic beads. Cpn60α1 and Cpn60β1–β3 were co-purified with both Cpn60β1 and Cpn60β4 (Tables 1 and S2). These results confirmed that Cpn60α1 and Cpn60β1–β4 form a heterooligomeric complex in vivo.

The ratio between protein emPAI scores can be used to estimate the relative amounts of protein in the different samples [40]. The emPAI ratios of Cpn60α1 and Cpn60β1–β3 detected in Cpn60β4- and Cpn60β1-purified samples were 3.9 and 0.47–1.26 (Cpn60β4/Cpn60β1), respectively, suggesting that comparable amounts of Cpn60 complexes were used for MS analysis. This estimation was confirmed by the similar intensity of the Cpn60 subunit bands detected by SDS-PAGE (Figure S5A). Interestingly, 24 peptides of an NDH subunit, NdhH, were found in the Cpn60β4-purified fraction. No other NDH subunits or NDH biogenesis factors were found in any sample other than the NdhJ detected in the Cpn60β1-purified extraction (Table 1). Although NdhH was also co-purified with Cpn60β1, only two NdhH peptides were detected (Table 1 and Figure S5B) and the emPAI ratio of NdhH from Cpn60β4- and Cpn60β1-purified samples was 43.4. Aside from the nonspecific proteins detected in WT as well as chaperonin subunits detected in Cpn60β4-IP sample, NdhH was the most abundant protein found in the Cpn60β4-purified sample (Table S2). These results indicate that the Cpn60 complex containing Cpn60β4 can specifically recognize unfolded NdhH. NdhH was also detected in the Cpn60β1-purified sample (Table 1), suggesting that Cpn60 complexes containing Cpn60β1 also can interact with NdhH. However, when Cpn60β1-HA was introduced into *crr27-1*, the transformation did not rescue NDH activity (Figures 1 and 2), suggesting that Cpn60 complexes lacking Cpn60β4 cannot produce native NdhH even though they can bind to it. This idea is consistent with the fact that *crr27* accumulates the band II subsupercomplex (Figure 2).

### Assembly of NDH Subcomplex A Is Impaired in *crr27*

Although the functional NDH complex is localized to the thylakoids, three assembly intermediate complexes including NdhH are present in the chloroplast stroma (Figure S6) [41]. Nuclear-encoded factors CRR6 and CRR7 may be required for integration of these intermediates into thylakoids to form the functional NDH complex. In *crr27-1*, the level of stroma-localized NdhH was significantly reduced (Figure S6A). Furthermore, 2D CN/SDS-PAGE and immunoblot studies showed that the accumulation of the 500 kDa and 400 kDa intermediate complexes was impaired in *crr27-1* (Figure S6B), implying that only NdhH folded by the Cpn60 complex including Cpn60β4 can be efficiently incorporated into these two assembly intermediates and further into thylakoids. These results also suggest that the folding of NdhH via the Cpn60 complex containing Cpn60β4 occurs at the initial step of NDH subcomplex A biogenesis.

### The Unique C-Terminus of Cpn60β4 Is Required for Its Specific Function

Based on a transcriptome database of *Arabidopsis*, ATTED-II [42], we found that the *Cpn60β4* gene, but not other *Cpn60* genes, is co-expressed with genes encoding NDH subunits and NDH biogenesis factors (Table S3). This pattern is consistent with our findings that Cpn60β4 is specifically required for the folding of NdhH. However, the question remains as to why the other Cpn60β proteins cannot complement the function of Cpn60β4.

The mycobacterial GroEL1 has a histidine-rich C-terminus that appears to be critical for its specific function in association with proteins required for bacterial biofilm formation [18]. Cpn60β4 also contains a C-terminal extension that is not conserved in other Cpn60β proteins (Figures 4A and S7). Although the C-terminus of Cpn60β4 is not conserved in plants, the region is rich in positively charged residues (Figure 4A). To study whether the C-terminus is important for Cpn60β4 function, HA-tagged Cpn60β4 lacking the C-terminus or exchanged by the short C-terminal tail of Cpn60β1 was expressed in *crr27-1* (Figure 4B). 2D CN/SDS-PAGE immunoblot analysis showed that the mutant versions of Cpn60β4 can be incorporated into the Cpn60 complex (Figure 4C), excluding the possibility that the C-terminus of Cpn60β4 is required for the stabilization or formation of the chaperonin complex. Although the levels of mutant Cpn60β4 were approximately twice those of the WT version of Cpn60β4 in the stroma, NdhH levels in thylakoids were reduced by approximately one half in the Cpn60β4-HA lines (Figure 4B), resulting in the reduction of NDH activity (Figure 4D). These results indicate that the folding efficiency of NdhH was reduced in the absence of the Cpn60β4-specific C-terminus.

**Figure 4:** C-terminal of Cpn60β4 is required for the Cpn60β4 function. (A) C-terminal alignment of Cpn60 subunits. Cpn60β4 from *Arabidopsis thaliana* (At), *Arabidopsis lyrata* (Al), *Oryza sativa* (Os), *Zea mays* (Zm), and *Populus trichocarpa* (Pt) were aligned with the *Arabidopsis* Cpn60β1–β3 and Cpn60α1 and the *E. coli* GroEL. Positions of the deletion and the C-terminal swapping are shown. The number of negatively (−) and positively (+) charged residues in the region is indicated. (B) Protein blot analysis of NdhH and Cpn60β4. RbcL and Cyt *f* were used as loading controls. The series of dilutions is indicated. (C) The C-terminus of Cpn60β4 is not essential for the assembly of the chaperonin complex. Stromal protein complexes isolated from *crr27-1* complemented by Cpn60β4 truncated in the C-terminus (Cpn60β4(-C)-HA) and from *crr27-1* transformed by Cpn60β4, in which the C-terminus was exchanged for that of Cpn60β1 (Cpn60β4(+β1C)-HA), were separated by CN-PAGE, followed by 2-D SDS-PAGE. The proteins were immunodetected with specific antibodies. A short arrow indicates the position of the Cpn60 complex. (D) NDH activity monitored by Chl florescence as in Figure 1B. *crr27-1+Cpn60β4-HA*, *crr27-1* transformed by WT genomic *Cpn60β4*; *crr27-1+Cpn60β4(-C)-HA*, *crr27-1* transformed by Cpn60β4 truncated in the C-terminus; *crr27-1+Cpn60β4(+β1C)-HA*, *crr27-1* transformed by Cpn60β4, in which the C-terminus was exchanged for that of Cpn60β1; *crr27-1+Cpn60β4(CM)-HA*, *crr27-1* transformed by Cpn60β4 containing the amino acid alterations in the wall of central cavity. All of the proteins were fused to the HA-epitope tag on their C-termini. (E) The net charge of each subunit wall exposed to the central cavity in the *cis* ring. As shown in Figure S7, the multiple charged residues, which are highly conserved among Cpn60β4 but not in Cpn60β1–β3 subunits, were altered in AtCpn60β4 to the corresponding amino acids in AtCpn60β1, resulting in a net charge of −4 (AtCpn60β4(CM)). (F) Immunoblot analysis of NdhH and Cpn60β4 from *crr27-1* expressing the AtCpn60β4(CM)-HA protein. (G) Protein blot analysis of NdhH and Cpn60β4. *crr27-1*+*Cpn60β4(ΔC+CM)-HA*, *crr27-1* transformed by a multiple mutant version of Cpn60β4 containing the amino acid alterations in the wall of central cavity (AtCpn60β4(CM)) and truncated in its C-terminus (Cpn60β4(-C)). The proteins were fused to the HA-tag on their C-termini. RbcL and Cyt *f* were used as loading controls and the series of dilutions is indicated.

In the absence of the C-terminal tail, NdhH is still partially assembled (Figure 5B). We also transformed *crr27* with Cpn60β1 fused with the Cpn60β4 C-terminal tail, but NdhH folding activity was not complemented (unpublished data). These results suggest that other features of Cpn60β4 are required for its specific function. Protein sequence alignment revealed that the ATP/ADP and Mg^2+^ binding sites are highly conserved between Cpn60β4 and the other three Cpn60β subunits (Figure S7), which is consistent with the fact that Cpn60β4 is an intrinsic subunit of the Cpn60 complex (Figure 3). However, the proposed substrate-binding residues are less conserved (Figure S7), which may explain why Cpn60β4 has a high affinity specifically for NdhH. Protein sequence alignment also showed that up to 31 amino acid residues are highly conserved among the putative Cpn60β4 orthologs, but their properties are different from the corresponding residues in other Cpn60β subunits (Figures S7 and S8). Three-dimensional (3-D) structure analyses mapped these residues to the apical, intermediate, and equatorial domains of the Cpn60β4 subunit (Figure S8).

**Figure 5:** Evolutionary analyses of the chloroplast Cpn60β4 subunits. (A) A phylogenetic tree of the chloroplast chaperonin 60 and cyanobacterial GroEL proteins. Chaperonin subunits from fully sequenced genomes of angiosperms (*Arabidopsis thaliana*, *Arabidopsis lyrata*, *Populus trichocarpa*, *Zea mays*, and *Oryza sativa*) and a bryophyte (*Physcomitrella patens*) were retrieved from GenBank or Phytozome (http://www.phytozome.net/). The GroEL sequences from *Synechocystis* SP. PCC 6803 and a Cpn60β sequence from *Marchantia polymorpha*, which is used to complement the *crr27-1* mutant in (B), are also included. The tree was generated using both Maximum-likelihood (ML) and Bayesian methods. ML and Bayesian consensus trees were topologically congruent and only ML topology is shown and drawn to scale. Numbers at each node in the ML tree signify bootstrap/posterior probability values (>50%) from ML and Bayesian methods, respectively. Support values less than 50 are shown as hyphens (−). The sequence alignments used to generate the ML and Bayesian tree are available in Dataset S1. Proteins highlighted with yellow boxes were investigated in this study. (B) Immunodetection of chloroplast proteins from WT, *crr27-1*, *crr27-1* complemented by AtCpn60β4-HA, and three lines of *crr27-1* complemented by MpCpn60β-HA (L1–L3).

Of the 31 conserved residues in Cpn60β4, several charged amino acids are located inside the cavity (Figure S8). The negatively charged GroEL cavity wall is required for rapid folding of some substrates [43]. In *E. coli*, each GroEL subunit has 27 negatively and 21 positively charged amino acids exposed to the central cavity in the *cis-*conformation, resulting in a net charge of −6 [44]. By analogy with *E. coli* GroEL, Cpn60α1 and Cpn60β1 have net charges of −4 and −6, respectively. However, Cpn60β4 in *Arabidopsis* has a more positive charge of 0, and this trend is found for Cpn60β4 in other plants (charges ranging from −2 to +2) (Figure 4E). To investigate the significance of the positively charged cavity wall in the folding of NdhH, the multiple charged residues, which are highly conserved in Cpn60β4 but not in Cpn60β1–β3 subunits, were converted to the corresponding amino acids of AtCpn60β1 and the mutant genes were introduced into *crr27-1* plants. The sites correspond to 5 out of 31 amino acid residues indicated in Figure S8. Although the mutant Cpn60β4 has a net charge of −4 (Figure 4E), NdhH level and NDH activity were fully rescued in the transformed plants (Figure 4D and 4F). We also transformed a version of Cpn60β4 with the amino acid alterations on the wall of the central cavity and the deletion of the C-terminus into *crr27-1*. In these lines, NdhH levels in thylakoids were reduced to ∼50% of the Cpn60β4-HA lines (Figure 4G), similar to the results in *crr27-1* transformed by Cpn60β4 lacking its C-terminus (Figure 4B). These results suggest that the positive charge of the cavity wall is not crucial for the folding of NdhH. The residues specifically conserved in the putative Cpn60β4 orthologs are dispersed throughout the molecule except for five positively charged sites facing the cavity wall (Figure S8), and it is not feasible to determine the sites responsible for the specific function by the site-directed mutagenesis. Proper folding of NdhH may require both the drastic alteration in the sequence as well as the C-terminal extension.

### Evolution of the Cpn60β4 Subunit

Both chloroplast Cpn60 and NDH complexes are thought to have originated from their cyanobacterial ancestors, GroEL2 [45] and NDH-1 [32]. NdhH is highly conserved in *Arabidopsis*, *Physcomitrella patens* (moss) and cyanobacteria (Figure S9). NdhH is a 45.5 kDa protein with α+β domains (Figure S9) [46], and theoretically it can be fully encapsulated within the chaperonin cage. In contrast to NdhH, the structure of Cpn60 is not conserved among organisms. To clarify the evolution and ancestry of Cpn60β subunits in plants, we compared the amino acid sequences of members in several fully sequenced genomes (Figure 5A). In addition to the distinct clades of Cpn60α and Cpn60β, Cpn60β proteins were further divided into two clades: putative AtCpn60β4 orthologs and other Cpn60β genes (major Cpn60β). The orthologs of AtCpn60β1–β3 were found in the closely related *Arabidopsis lyrata*, but two major Cpn60β proteins of poplar (*Populus trichocarpa*) were related only to AtCpn60β3. In contrast, the major Cpn60β subunits of monocots form a different subclade, and maize (*Zea mays*) and rice (*Oryza sativa*) each contain two major Cpn60β subunits (Figure 5A). These facts suggest that gene duplication of major Cpn60β subunit genes took place independently both in monocots and eudicots. In contrast, a single copy of the putative Cpn60β4 ortholog was detected in angiosperms (Figure 5A).

A total of three Cpn60β subunits were found in *Physcomitrella patens* and they are related to major Cpn60β subunits in angiosperms (Figure 5A). Notably, no ortholog of Cpn60β4 was found in *P. patens*. The phylogenetic tree indicates that the origin of Cpn60β4 can be traced to the origin of land plants and that Cpn60β4 was lost in the descendent lineage of bryophytes. Due to the low bootstrap support of the evolutionary relationships between angiosperm and bryophyte major Cpn60β subunits (72/0.90 as shown in Figure 5), it is also likely that the Cpn60β4 orthologs were produced by a gene duplication event that took place only in a common ancestor of angiosperms and underwent a rapid rate of evolution to obtain the novel function. In any case, *P. patens* should use a different mechanism to assist the folding of NdhH, as it also contains the chloroplast NDH complex.

To study whether the Cpn60β subunits in bryophytes can facilitate the folding of NdhH, we introduced the *Cpn60β* gene isolated from liverwort (*Marchantia polymorpha*) into *crr27-1* (Figure 5B). We identified only one gene copy encoding Cpn60β in *M. polymorpha*, possibly due to incomplete genome information. Immunoblots detected a trace amount of NdhH in the thylakoids of three transgenic lines, although the levels of MpCpn60β were comparable to those of AtCpn60β4 in *crr27-1* transformed by *AtCpn60β4-HA* (Figure 5B), suggesting that MpCpn60β partially rescues the phenotype of *crr27-1* and that Cpn60β in bryophytes retains its ability in assisting the folding of NdhH. As MpCpn60β forms the heterologous Cpn60 complex with AtCpn60α, we could not compare the efficiency of the NdhH folding with the complex including AtCpn60β.

## Discussion

Although multiple chaperonin genes are present in a significant proportion of bacteria and eukaryotes, the function and biological significance of this kind of divergent evolution have yet to be revealed [13]. Generally, it is thought that the major subunits fulfill the housekeeping chaperonin function. The minor chaperonin subunits may increase the general chaperoning ability by elevating the chaperonin abundance in response to different environmental conditions. In this study, we demonstrated that the highly divergent chloroplast chaperonin subunit Cpn60β4 is specifically and strictly required for the folding of the NDH subunit NdhH.

Although Cpn60β4 is highly divergent from the major Cpn60β subunits (Figure 5), it is an intrinsic chaperonin subunit and forms a heterooligomeric Cpn60 complex with Cpn60α1 and other Cpn60β subunits (Figure 3 and Table 1), suggesting the involvement of this specific Cpn60 complex in assisting the folding of some proteins. In line with this idea and the *crr27* phenotype, the NDH subunit NdhH was copurified with the heterooligomeric Cpn60 complex including Cpn60β4 (Table 1). Although the Cpn60 complex lacking Cpn60β4 also interacts with NdhH with less affinity (Tables 1 and S2), it cannot produce native NdhH for further NDH complex assembly (Figures 1 and 2), implying that Cpn60β4 is required for both high-affinity binding and folding of NdhH. In contrast with the observation in *R. meliloti*, *B. japonicum*, and *R. leguminosarum* [15]–[17], in which the function of the unusual chaperonins can be partially replaced by other chaperonins, Cpn60β4 is absolutely required for the folding of NdhH. These data support the proposal that multiple chaperonin subunits have evolved to assist the folding of specific proteins, although the functional specialization is not absolute in some cases.

What is the structural basis for the functional specialization of Cpn60β4? We clarified that the unusual C-terminus of Cpn60β4 is required for the full activity of the Cpn60 complex containing Cpn60β4 for folding NdhH. The aforementioned GroEL1 protein in *M*. *smegmatis* also has an unusual histidine-rich C-terminus, which was shown to be essential for the specific function of GroEL1 [18]. These observations suggest that modification of the C-terminus is necessary to facilitate the folding of specific targets. This idea is consistent with the fact that the many bacterial genomes encode an additional chaperonin with an unusual C-terminus [13].

The C-terminus of Cpn60β4 is not required for the formation of the specific chaperonin complex containing Cpn60β4 (Figure 4C). Thus, it should have some special functions in other steps during the folding of NdhH. The chaperonin complex containing Cpn60β4 and its substrate NdhH can be purified via the HA tag fused with the C-terminus of Cpn60β4 (Table 1 and Figure 3C). As the *cis* ring is capped by a co-chaperone, it is likely that the C-terminal tail of Cpn60β4 extends from the *trans* ring so that the chaperonin complex containing Cpn60β4 can be trapped by microbeads coupled with HA antibody. Alternatively, the chaperonin complex was purified by the C-terminal tail extruding from the *cis* ring, which was not capped but already associated with the substrate NdhH. The protruded C-terminal tail of Cpn60β4 might promote the high affinity binding with NdhH, ensuring that the nonnative NdhH can be efficiently captured by the Cpn60 complex containing Cpn60β4. In addition, enclosure of the nonnative NdhH protein inside the cavity by a co-chaperonin will lead to the encapsulation of the C-terminus. Consequently, the C-terminus might also contribute to the specific function of Cpn60β4 in assisting the folding of NdhH in the cavity. It has been reported that changing the length of the C-terminus of GroEL can affect the folding speed of some substrates [43],[47]. Farr et al. provided further evidence that the elongated C-terminus perturbed the ATPase activity, and the disturbance of the rate of ATP hydrolysis resulted in the modification of the folding rate of some substrates [48]. The physical properties of the C-terminus [49] such as the length [43],[47], hydrophilicity [50], and hydrophobicity [43] have been proposed to be critical for the substrate folding in the cavity. We also found that the C-terminus of the Cpn60β4 is rich in positively charged residues (Figure 4A). Thus, it is likely that these unusual C-termini provide specific environments in the chaperonin cavity and/or modify the chaperonin ATPase rate of the chaperonin complex.

The deletion of up to 27 residues of the C-terminal tail of GroEL does not affect the growth of *E. coli* [51],[52], suggesting that the C-terminal motif does not play an essential role in assisting the folding of substrates. It is also true that Cpn60β4 lacking its unusual C-terminal tail still can partially assist the folding of NdhH (Figure 4B). Our results showed that the charged residues exposed on the cavity wall do not play a critical role for the specific function (Figure 4F). In addition, we discovered many residues that are potentially important for the specific function of Cpn60β4 (Figures S7 and S8). Among them, several residues are mapped to the intermediate domain or near the ATP/ADP binding site (Figure S8). The *E. coli* GroEL with specific mutations in this region can improve the folding activity for green fluorescent protein (GFP), most likely through the adjustment of the ATPase activity [53]. Recently, the apical domain of GroEL1 from *Mycobacterium tuberculosis* was shown to be sufficient for binding the specific substrate KasA [54]. Notably, some residues are specifically conserved in the apical domain of the putative Cpn60β4 orthologs (Figure S8). In addition, other conserved residues in AtCpn60β4 orthologs may be required for the formation of the Cpn60 complex including Cpn60β4 with certain stoichiometry or to provide certain physical features of the cavity wall. With the exception of the C-terminal extension, we could not specify the residues that are required for Cpn60β4 function. It is likely that some residues that are specifically conserved in the putative Cpn60β4 orthologs cumulatively contribute to their specific function, and this drastic evolution may have been necessary to assist the folding of NdhH. However, it is puzzling that MpCpn60β, which is related to the major AtCpn60β subunits, partly complemented the function of Cpn60β4 and that bryophytes do not contain the Cpn60β4 orthlogs (Figure 5).

Specific mutations of GroEL can improve the folding activity of a specific protein [53]. However, mutated GroEL has a reduced ability to fold a variety of natural substrates, suggesting a conflict between the specific ability of GroEL to fold particular substrates and its general ability in assisting the folding of a wide range of substrates [53]. By combining all of the features acquired during the evolution of plants, Cpn60β4 allows the Cpn60 complex to assist the folding of the specific substrate, NdhH. However, other Cpn60 subunits, especially the major Cpn60β proteins, may have become optimized to support the efficient folding of other obligate substrates. Through this kind of divergent evolution, the chaperonin system can resolve the apparent conflict between specialization and generalization of its function.

## Materials and Methods

### Plant Material and Growth Conditions

*Arabidopsis thaliana* (ecotypes Col-0 and Nössen) plants were grown in a growth chamber (50 µmol photons m^−2^ s^−1^, 16 h photoperiod, 23°C) for 3 to 4 wk. *cpn60α1* was mutagenized by ethyl methanesulfonate [55]. *crr27-3* (ecotypes Nössen) was isolated from a collection of *Ds* transposon insertion lines [36]. *crr27-1* (SALK_136518, Col-0) and *crr27-2* (SALK_064887, Col-0) were obtained from the ABRC Stock Center. For complementation experiments, vectors were transferred into *Agrobacterium tumefaciens* C58C by electroporation, and the bacteria were used to transform *crr27-1* by floral dipping.

### Chlorophyll Fluorescence Analysis

Chlorophyll fluorescence was measured using a MINI-PAM (pulse amplitude modulation) portable chlorophyll fluorometer (Walz, Effeltrich, Germany). The transient increase in chlorophyll fluorescence after turning off AL was monitored as previously described [33]. Leaves were exposed to AL (50 µmol photons m^−2^ s^−1^) for 5 min. AL was turned off and the subsequent transient rise in fluorescence ascribed to NDH activity was monitored. Fluorescence levels were standardized to the maximum fluorescence levels of closed PSII (*Fm*) by applying saturating-light pulses (SP).

To investigate the light intensity dependence of two chlorophyll fluorescence parameters, ETR and NPQ, measuring light (650 nm, 0.1 µmol photons m^−2^ s^−1^) was used to excite the minimum fluorescence at open PSII centers in the dark-adapted state (*F_o_*). A saturating pulse of white light (800 ms, 8,000 µmol photons m^−2^ s^−1^) was applied to determine the maximum fluorescence at closed PSII centers in the dark (*Fm*) or during light illumination (*Fm’*). The steady-state fluorescence level (*Fs*) was recorded during AL illumination (15–1,000 µmol photons m^−2^ s^−1^). These photosynthetic parameters were recoded 2 min after the change of AL intensity. Φ_PSII_ was calculated as (*Fm′* – *Fs*)/*Fm′*. ETR and NPQ were calculated as Φ_PSII_×photon flux density (µmol photons m^−2^ s^−1^) and (*Fm* – *Fm′*)/*Fm′*, respectively.

### Thylakoid Membrane Isolation, BN-PAGE, CN-PAGE, and Immunoblot Analysis

Freshly isolated chloroplasts were osmotically ruptured in buffer containing 20 mM HEPES–KOH (pH 7.6), 5 mM MgCl_2_, and 2.5 mM EDTA. Thylakoid membranes were separated from the stromal fraction by centrifugation (17,000 g for 10 min at 4°C). CN-PAGE, BN-PAGE, and 2-D CN/SDS-PAGE were performed according to previous reports [27],[38]. For immunoblot analysis, thylakoid and stromal proteins were loaded by equal chlorophyll and protein content, respectively. The stromal protein contents were determined with a Bio-Rad Protein Assay Kit (cat. No. 500-0006). Immunoblot signals were detected with an ECL plus Western Blotting Detection Kit (GE Healthcare) and visualized with a Luminescent image analyzer (LAS)-3000 (Fuji Film). Immunoblots were quantified by Imagemaster software (Amersham Pharmacia Biotech).

### RNA Isolation and RT-PCR Analysis

Total RNA was isolated from *Arabidopsis* leaves with an RNeasy Plant Mini Kit (Qiagen) and treated with DNase I (Invitrogen). Total RNA (5 µg) was reverse transcribed using the SuperScript III First-Strand Synthesis System (Invitrogen) in a total volume of 20 µl. The cDNA was used in 35 cycles of PCR with the following primers: 5′-TGGCTCTGTCACCAAGAAGCTTCAG-3′ and 5′-GCTTTCTGGGTGAATCCGTTGGTAA-3′. RT-PCR products were separated on agarose gels and detected by ethidium bromide staining.

### Affinity Chromatography of the Chaperonin-Substrate Complexes

Cpn60-substrate complexes were isolated from *crr27-1* plants expressing HA-tagged Cpn60β subunits with the µMACS HA isolation kit under the conditions previously established [11], with a minor modification. Freshly isolated chloroplasts were osmotically ruptured in lysis buffer (50 mM Tris-HCl pH 8.0, 0.01% Tween 20, 10 mM MgCl_2_, 20 mM glucose, 20 U/ml hexokinase) plus protease inhibitors (Complete mini, Roche). Within 10 s after lysis, ADP was added to a final concentration of 10 mM. Thylakoid membranes were pelleted by centrifugation at 20,000 g for 10 min at 4°C and the supernatants were transferred to new tubes. NaCl was added to the supernatants to a final concentration of 150 mM and then mixed with 50 µl anti-HA MicroBeads (Miltenyi Biotec.). After incubation for 2 h at 4°C, the beads were transferred to columns placed in a magnetic field. Columns were rinsed four times with 200 µl washing buffer I (50 mM Tris-HCl pH 8.0, 1% Triton, 0.5% Sodium deoxycholate, 150 mM NaCl, 5 mM ADP) and twice with 200 µl washing buffer II (50 mM Tris-HCl pH 8.0, 1% Triton, 150 mM NaCl, 5 mM ADP). After final washing with 200 µl washing buffer III (25 mM Tris-HCl pH 7.5, 5 mM ADP), the chaperonin-substrate complex was eluted with elution buffer (50 mM Tris-HCl pH 6.8, 50 mM DTT, 1% SDS, 1 mM EDTA, 0.005% bromophenol blue, 10% glycerol). Total protein was separated on 12.5% SDS-PAGE gels (Perfect NT Gel, DRC) and stained with CBB. SDS-PAGE lanes were cut into four slices and analyzed by LC-MS/MS analyses.

### Mass Spectrometric Analysis and Database Searching

Peptide Preparation and LC-MS/MS analyses were performed as previously described [39]. The excised bands were treated twice with 25 mM ammonium bicarbonate in 30% (v/v) acetonitrile for 10 min and 100% (v/v) acetonitrile for 15 min, and then dried in a vacuum concentrator. The dried gel pieces were treated with 0.01 mg/ml trypsin (sequence grade; Promega)/50 mM ammonium bicarbonate and incubated at 37°C for 16 h. The digested peptides were recovered twice with 20 µl 5% (v/v) formic acid/50% (v/v) acetonitrile. The extracted peptides were combined and then dried in a vacuum concentrator. LC-MS/MS analyses were performed on an LTQ-Orbitrap XL-HTC-PAL system. MS/MS spectra were compared by the MASCOT server (v. 2.2) against TAIR8 (The Arabidopsis Information Resource) with the following search parameters: set-off threshold at 0.05 in the ion-score cut-off; peptide tolerance, 10 ppm; MS/MS tolerance, ±0.8 Da; peptide charge, 2+ or 3+; trypsin as enzyme allowing up to one missed cleavage; carboxymethylation on cysteines as a fixed modification; and oxidation on methionine as a variable modification.

### Phylogenetic Analysis

Chaperonin protein sequences were first aligned using the CLUSTALX 1.83 program [56]. The protein alignment was further refined manually and 534 conserved sites were used for phylogenetic analysis. Phylogenetic trees were constructed by using both the maximum likelihood (ML) and Bayesian methods to ensure the robustness of our analysis. ML trees were constructed by using PHYML version 2.4 [57] with WAG model selected via MODELTEST 3.06 [58], and support for each branch was assessed using bootstrap analyses with 100 bootstrap replicates. Bayesian trees were constructed using MrBayes software [59] with the WAG model. Four chains of Markov chain Monte Carlo were run, sampling one tree every 1,000 generations for 1,000,000 generations, starting with a random tree. The first 50,000 generations were excluded as burn-in to ensure that the chains reached stationary. The posterior probability was used to estimate nodal robustness.

### Homology Modeling

The structure model of the Cpn60β4 protein was obtained by homology modeling using the SWISS-MODEL server (http://swissmodel.expasy.org/) [60], and the crystal structure of *E. coli* GroEL (PDB 1AON, Chain A) was used as a modeling template. The 3-D predicted structure was visualized using the PyMol software.

### Accession Numbers

Sequence data from this article can be found in the Arabidopsis Genome Initiative or GenBank/EMBL databases under the following accession numbers: At (*Arabidopsis thaliana*) Cpn60α1 (At2g28000), AtCpn60α2 (At5g18820), AtCpn60β1 (At1g55490), AtCpn60β2 (At3g13470), AtCpn60β3 (At5g56500), AtCpn60β4 (At1g26230), AtNdhH (BAA84443), Al (*Arabidopsis lyrata*) Cpn60α1 (481708), AlCpn60α2 (488768), AlCpn60β1 (474606), AlCpn60β3 (495739), AlCpn60β4 (890123), Sy (*Synechocystis* SP. PCC 6803) GroEL-1 (NP_440731), SyGroEL-2 (NP_442170), SyNdhH (CAA43057), GroEL (*Escherichia coli*) (NP_418567), and Pp (*Physcomitrella patens*) NdhH (BAC85094).

## Supporting Information

Figure S1 Protein blot analysis of chloroplast proteins. Equal amounts of total protein extracted from the leaves of WT, *cpn60α1*, and *crr27-1* plants were separated by SDS-PAGE and immunodetected by antibodies against stromal proteins Cpn60α, Cpn60β, and RbcL (A) or thylakoid proteins NdhH, NDH18, NDF1, FKBP16-2, PsaA, Cyt *f*, D1, and LHCII (B), which represent the thylakoid protein complexes indicated.
(TIF)

Figure S2 In vivo analysis of electron transport activity. (A) Light-intensity dependence of ETR. ETR is depicted relative to the maximum value of Φ_PSII_ × light intensity (μmol photons m^−2^ s^−1^) in the WT (100%). (B) Light-intensity dependence of NPQ of chlorophyll fluorescence. All values represent the mean ± SD (*n* = 5) in (A) and (B).
(TIF)

Figure S3 Analysis of thylakoid and stromal protein complexes by native PAGE. (A) Freshly isolated thylakoid membranes from WT (ecotype Col-0 and Nössen), *crr27*, and *ndhl* plants were solubilized in 1% *n*-dodecyl-β-d-maltoside (DM) at a chlorophyll concentration of 1 µg μl^−1^, and the protein sample was separated by 5%–12% BN-PAGE. The major protein complexes were assigned based on a previous report [39]. Band I, NDH-PSI supercomplex detected in WT; Band II, sub-NDH-PSI supercomplex detected in the *crr27* and *ndhl* mutants. (B) Stromal protein complexes isolated from WT and *crr27-1* plants were separated by CN-PAGE followed by 2-dimensional SDS-PAGE. After electrophoresis, protein was stained with CBB. The positions of the molecular markers are indicated above the gel. The Cpn60 complex was assigned on the basis of a previous report [27].
(TIFF)

Figure S4 Detection of Cpn60β4 in WT plants. (A) CN-PAGE analysis of stromal protein complexes isolated from WT plants. After electrophoresis, the CN-gel was stained with CBB. The protein band corresponding to the position of the Cpn60 complex (the boxed area indicated by an arrow) was excised from the gel and analyzed by LC-MS/MS analysis. (B) Summary of the chaperonin subunits detected in the excised band. (C) The peptides of Cpn60β4 detected in the excised band by MS analysis. Total proteins detected are listed in Table S1.
(TIFF)

Figure S5 Immunoaffinity purification of Cpn60-substrate complexes. (A) Chaperonin complexes containing Cpn60β1 and Cpn60β4 subunits were purified from *crr27-1* mutants expressing HA-tagged Cpn60β1 and Cpn60β4, respectively. After elution, total proteins were separated by SDS-PAGE and stained with CBB. Due to the low abundance of Cpn60β4, more stromal proteins were used for the purification, leading to an increase in non-specific binding of some proteins. Lanes were cut into four slices and total protein was analyzed by LC-MS/MS analysis. CK, WT plants without any transformation were used as a negative control. (B) NdhH peptides detected from the chaperonin complexes containing Cpn60β1 (upper) and Cpn60β4 (bottom) are indicated in red bold.
(TIFF)

Figure S6 Analysis of stromal protein complexes isolated from wild-type and *crr27-1* plants. (A) Immunodetection of NdhH isolated from the stroma of wild type (WT), *crr27-1*, *ndhl*, and *crr27-1* plants complemented with Cpn60β4. Equal amounts of stromal protein (8 µg) were loaded onto each well. WT thylakoid proteins corresponding to 2.5 µg chlorophyll were also analyzed. RbcL was used as a loading control. An asterisk represents non-specific signals. (B) Stromal protein complexes isolated from WT and *crr27-1* plants were separated by CN-PAGE followed by 2-dimensional SDS-PAGE. The proteins were immunodetected with specific antibodies against NdhH and RbcL. Vertical arrows indicate the positions of three assembly intermediates, which include NdhH.
(TIF)

Figure S7 Protein alignment of the mature chaperonin proteins. The origin of all chaperonin subunits is shown in Figure 5. GroEL from *E. coli* was also included in the alignment. Residues involved in ATP/ADP and Mg^2+^ binding are marked with +. Red and blue sharps (#) represent the residues for the substrate binding proposed by Fenton et al. [61] and Buckle et al. [62], respectively. The charged residues exposed to the central cavity in the *cis* ring are labeled with asterisks. The residues marked with red asterisks were selected for introducing the mutations as shown in Figure 4F. Amino acid residues that are highly conserved in the putative Cpn60β4 orthologs and with different properties from the corresponding residues in major Cpn60β subunits are marked with solid red circles under the protein sequences. These residues were also highlighted as spheres in the structure model of Cpn60β4 in Figure S8. The amino acid mutated in the *cpn60α1* mutant is labeled with a triangle. Positions of the deletion and the C-terminal swapping are shown.
(TIFF)

Figure S8 Predicted structure of the *Arabidopsis* Cpn60β4 subunit. A 3-dimensional (3D) structural model of *Arabidopsis* Cpn60β4 was generated with the Swiss Model alignment server. The structure model of *E. coli* GroEL (PDB 1AON, Chain A) was used as a modeling template. Predicted 3-D structure was displayed by using the PyMOL software. The apical domain (Ap), intermediate domain (Int), and equatorial domain (Eq) are shown in cyan, green, and blue, respectively. Highly conserved ATP/ADP and Mg^2+^ binding sites are marked with magenta spheres. Residues that are highly conserved in Cpn60β4 subunits but exhibit different properties with the corresponding residues in other Cpn60β are highlighted with yellow and red spheres. Among them, sites marked with red, blue, and cyan arrows represent residues near the ATP binding site or in the intermediate domain, residues exposed to the central cavity in the *cis*-conformation of the chaperonin complex, and one residue involved in the substrate binding, respectively. Sites marked with red spheres (indicated with green arrows) were selected for introducing the mutations shown in Figure 4F.
(TIFF)

Figure S9 Structure and evolution of NdhH. (A) Ribbon models of the Complex I Subunit Nqo4 (PDB 2fugV) from *Thermus thermophilus*. Nqo4 corresponds to NdhH in the chloroplast NDH complex. (B) A predicted structure of the *Arabidopsis* NdhH. Homology models were generated with the Swiss Model alignment server. The α-helix is shown in red, β-sheet in blue, and other domains in yellow. (C) Protein alignment of the NdhH subunits from *Arabidopsis thaliana* (AtNdhH), *Physcomitrella patens* (PpNdhH), and *Synechocystis* SP. PCC 6803 (SyNdhH).
(TIFF)

Table S1 Total protein detected in the excised band corresponding to the Cpn60 complex in CN-gel.
(XLS)

Table S2 Total protein detected in the WT-IP, Cpn60β1-IP, and Cpn60β4-IP fractions.
(XLS)

Table S3 *r* value between *Cpn60β4* and *Cpn60α1* with NDH complex-related or chaperonin subunit genes.
(DOC)

Dataset S1 Protein sequences used for alignment and phylogenetic tree construction.
(DOC)

## Abbreviations

AL: actinic light
BN-PAGE: blue native PAGE
CN-PAGE: clear native PAGE
*crr*: *chlororespiratory reduction*
Cyt: cytochrome
emPAI: exponentially modified Protein Abundance Index
HA: influenza hemagglutinin protein epitope
LC-MS/MS: liquid chromatography-tandem mass spectrometry
NDH: NADH dehydrogenase-like complex
PAM: pulse amplitude modulation fluorometry
PQ: plastoquinone
PSI: photosystem I
PSII: photosystem II
WT: wild type
